# Segmentation of Brain Tissues from MRI Images Using Multitask Fuzzy Clustering Algorithm

**DOI:** 10.1155/2023/4387134

**Published:** 2023-02-17

**Authors:** Yunlan Zhao, Zhiyong Huang, Hangjun Che, Fang Xie, Man Liu, Mengyao Wang, Daming Sun

**Affiliations:** ^1^School of Microelectronics and Communication Engineering, Chongqing University, Chongqing 400044, China; ^2^School of Electronics and Information Engineering, Southwest University, Chongqing 400715, China; ^3^Chongqing Engineering Research Center of Medical Electronics and Information Technology, Chongqing University of Posts and Telecommunications, Chongqing 400065, China

## Abstract

In recent years, brain magnetic resonance imaging (MRI) image segmentation has drawn considerable attention. MRI image segmentation result provides a basis for medical diagnosis. The segmentation result influences the clinical treatment directly. Nevertheless, MRI images have shortcomings such as noise and the inhomogeneity of grayscale. The performance of traditional segmentation algorithms still needs further improvement. In this paper, we propose a novel brain MRI image segmentation algorithm based on fuzzy C-means (FCM) clustering algorithm to improve the segmentation accuracy. First, we introduce multitask learning strategy into FCM to extract public information among different segmentation tasks. It combines the advantages of the two algorithms. The algorithm enables to utilize both public information among different tasks and individual information within tasks. Then, we design an adaptive task weight learning mechanism, and a weighted multitask fuzzy C-means (WMT-FCM) clustering algorithm is proposed. Under the adaptive task weight learning mechanism, each task obtains the optimal weight and achieves better clustering performance. Simulated MRI images from McConnell BrainWeb have been used to evaluate the proposed algorithm. Experimental results demonstrate that the proposed method provides more accurate and stable segmentation results than its competitors on the MRI images with various noise and intensity inhomogeneity.

## 1. Introduction

With the increasing demand for medical services, medical imaging technology continues to be improved. Technology plays a major role in computer-assisted medicine. There are multimodal medical imaging technologies, such as magnetic resonance imaging (MRI), positron emission tomography (PET) scanning, and computed tomography (CT) scanning. MRI has the advantages of a high data rate, no radiation, and high soft-tissue contrast [1]. MRI is generally used to visualize the structure and tissue of a patient [2].

With the great number of medical images increasing in number, manual interpretation of image information becomes an impossible challenge. Experts have different experiences and knowledge. It is impossible to obtain uniform and precise segmentation results [3]. Computer-assisted medical image processing plays a more and more important role. Image segmentation is an indispensable part of medical image processing [4]. The different tissues classification of the image provides a reference for doctors in disease diagnosis and intervention decisions. It helps improve diagnostic accuracy and efficiency. Hence, the research has great clinical significance in medical image segmentation.

Traditional image segmentation methods are divided into distinct categories according to their principles, such as threshold, clustering, region-based, and edge-based methods [5]. The fuzzy C-means (FCM) algorithm was first proposed by Bezdek et al. [6]. The FCM is widely used owing to its applicability and simplicity [7]. The FCM algorithm provides the ability to describe the fuzziness of the images. Therefore, the fuzzy clustering algorithm is appropriate for MRI images. Nevertheless, the performance of traditional FCM still needs further improvement [8]. The core problem is sensitive to noise and the initialization of cluster centroids in brain MRI image segmentation. To solve the problem, many improved FCM algorithms have been proposed. Enhancements have been tried to improve algorithm performance by introducing local spatial information [7, 9], integrating bioinspired algorithms [10–12], and enhancing the image [13]. Ji et al. [9] introduced a method called RSCFCM for brain MRI image segmentation by introducing a factor for the spatial direction to deal with noise. The algorithm improved the segmentation accuracy. Meena Prakash et al. [14] employed a brain MRI segmentation algorithm integrated with spatial information and contrast enhancement based on FCM, but the clustering performance of the algorithm is not much improved compared with the original FCM algorithm. Pham et al. [7] integrated the PSO algorithm and kernelized fuzzy entropy clustering with spatial information and bias correction algorithm, called the PSO-KFECSB algorithm, which improved the robustness to noise and initializations, but the computational cost of the algorithm increased. Vinurajkumar and Anandhavelu [13] proposed an enhanced fuzzy segmentation framework for extracting white matter, which exhibited low values of computational time, but the segmentation results are sensitive to the initialization of the fuzzy partition matrix.

MRI images of different subjects have much common information. The related information could improve the segmentation performance. Classical FCM only deals with a single task. The algorithm pays no attention to the related tasks and only utilizes limited information [15]. To overcome the limitation, many multitask-related algorithms have been proposed, such as transfer-learning clustering algorithms [16], multitask clustering algorithms [15, 17, 18], multiview clustering algorithms [3, 19], collaborative clustering algorithms [20], and subspace clustering algorithms. Multitask learning learns related tasks simultaneously and shares useful information, such as representation and parameters among related tasks. Multitask learning strategy improves the clustering performance and obtains higher accuracy [21]. Hua et al. [3] designed a multiview fuzzy clustering algorithm to extract multiple feature data from the original image. Experimental results prove that the segmentation method optimizes the segmentation effect. Jiang et al. [18] proposed a distributed multitask fuzzy C-means (DMFCM) clustering algorithm for MRI image segmentation, which can extract common and individual information among different clustering tasks. The public cluster centroids represent the common information of different tasks. DMFCM significantly outperforms traditional FCM. However, because the common information is obtained directly from the original pixel data, the computational complexity greatly increases.

Generally, the current brain MRI image segmentation algorithms suffer from the shortcomings such as the sensitivity to the cluster initialization, lack of robustness to noise, and high computational complexity. In this study, a new fuzzy clustering algorithm is to be explored for better improvement of the aforementioned problems. Based on the traditional FCM algorithm, we integrate multitask learning strategy and propose a weighted multitask fuzzy C-means clustering algorithm (WMT-FCM). WMT-FCM learns multiple different but related tasks simultaneously to extract public information. By introducing the adaptive weight learning mechanism, tasks are assigned optimal weights and can be adaptively learned to achieve a better clustering effect.

The summary of contributions in this research is as follows:

1. We integrate the traditional FCM algorithm and multitask learning strategy with a new objective function and propose an improved fuzzy clustering method to enhance the accuracy of brain MRI image segmentation.
2. We design an adaptive weight learning mechanism to obtain optimal weights for all tasks. Under the weight mechanism, the public information extracted from different tasks is more accurate, and each task can achieve better clustering effects.
3. We regard the public cluster centroids as the public information of different tasks. Taking into account a large amount of pixel data in the images, we capture public information from cluster centroids instead of raw pixel data. It contributes to reducing computational complexity.

## 2. Related Work

### 2.1. Fuzzy *C*-Means Algorithm

In 1965, Zadeh published a paper on fuzzy sets. This paper used “Fuzzy” to describe the uncertainty of the classification. A membership function was proposed to indicate the fuzzy degree of elements [22]. Compared with classical set theory, elements in fuzzy sets have no strict boundaries. In fuzzy theory, elements are assigned membership values instead of clear categories.

Bezdek et al. introduced fuzzy theory the into hard C-means (HCM) algorithm and proposed FCM [6]. The FCM algorithm divides targets into numerous subcategories according to the uncertainty. The idea of FCM is to assign each data instance to all clusters with membership values [23, 24]. It is an unsupervised fuzzy clustering algorithm with no requirement for human intervention in the implementation of the algorithm [25]. In addition, there is no requirement for setting a threshold in advance. HCM is a hard partitioning method, and the result is either 1 or 0. Compared with HCM, FCM is more suitable for dealing with fuzzy and uncertain problems [26].

The fuzzy clustering algorithm is widely applied to medical image processing. Militello et al. [27] proposed a semiautomated and interactive approach based on the spatial fuzzy C-means algorithm to segment masses on dynamic contrast-enhanced breast MRI. Al-Saeed et al. [28] proposed a fast-generalized fuzzy C-means algorithm and used the unsupervised algorithm to segment the liver from the rest of the abdomen organs on CT scans. Zhao et al. [29] integrated a deep belief network and FCM unsupervised deep clustering for lung cancer patient classification from lung CT images. Militello et al. [30] applied FCM to enhance automatic cell colony detection. Navaei Lavasani et al. [31] used the fuzzy C-means algorithm to segment prostate lesions on prostate dynamic contrast-enhanced MRI and obtained the diagnostic credibility increase. Rundo et al. [32] integrated T1w and T2w MRI image structural information based on the fuzzy C-means algorithm to enhance prostate gland segmentation.

Table 1 shows the symbols used in the FCM algorithm. Assume the input dataset with *N* data instances is **X**={*x*_1_, *x*_2_,……*x*_*N*_}, **V**={*v*_1_, *v*_2_,……*v*_*C*_} is the cluster center vector, **U**=[*u*_*ij*_]_*C*×*N*_ is the membership matrix, *u*_*ij*_ is the membership value of the *i*th data sample to the *j*th cluster, and *C*(1 < *C* < *N*) is the number of subcategories. The objective function of the FCM algorithm [6] is as follows:

(1) $$\begin{array}{c} J_{FCM}=\overset{N}{\underset{i=1}{\sum }}\overset{C}{\underset{j=1}{\sum }}u_{ij}^{m}{\left\|x_{i}-v_{j}\right\|}^{2}\text{.} \end{array}$$

Regarding the objective function *J*_FCM_, the constant *m* (*m* > 1) indicates the degree of ambiguity. When the value of *m* is larger, the fuzziness of clustering is higher. Therefore, a large value is not conducive to reduce the fuzziness. When the value of *m* equals 1, it is equivalent to the clustering result of the HCM algorithm. Usually, the value of *m* is assigned to 2 [2, 3, 24]. ‖*x*_*i*_ − *v*_*i*_‖^2^ is the Euclidean distance between data sample *x*_*i*_ and cluster *v*_*j*_. The constraints of the membership value are as follows:

(2) $$\begin{array}{c} \overset{C}{\underset{j=1}{\sum }}u_{ij}=1,0\leq \overset{N}{\underset{i=1}{\sum }}u_{ij}\leq N,u_{ij}\in \left[0,1\right]\text{.} \end{array}$$

The FCM algorithm minimizes the objective function by iteratively calculating the membership degree and cluster centers. The Lagrange multiplier method is used to solve the objective function. The cluster centers and membership values can be iteratively updated by the following equations:

(3) $$\begin{array}{c} u_{ij}=\frac{{\left({\left\|x_{i}-v_{j}\right\|}^{2}\right)}^{-1/m-1}}{\sum_{l=1}^{C}{\left({\left\|x_{i}-v_{j}\right\|}^{2}\right)}^{-1/m-1}}\text{,} \end{array}$$

(4) $$\begin{array}{c} v_{j}=\frac{\sum_{i=1}^{N}u_{ij}^{m}x_{i}}{\sum_{i=1}^{N}u_{ij}^{m}}\text{.} \end{array}$$

Considering the uncertainty and unclearness of brain tissue boundaries, the fuzzy clustering algorithm can be employed in image segmentation. The input dataset **X**={*x*_1_, *x*_2_,……*x*_*N*_} is the image pixel dataset, where *x*_*i*_ represents the grayscale of the *i*th pixel of the image. The segmentation of images is transformed into a clustering problem. That is, dividing *N* pixels into *C* cluster centers according to the final membership matrix.

The steps of segmentation images using the FCM algorithm are summarized as follows: (1) set the iteration stop threshold *ε*, the number of clusters *C*, fuzzy index *m*; (2) initialize the cluster centers randomly; (3) update the membership matrix and cluster centers according to equations (3) and (4); (4). Calculate the objective function; (5) If the objective function value converges, the algorithm stops, otherwise, it goes to step 3).

### 2.2. Multitask Learning Strategy

Multitask learning refers to performing multiple related tasks at the same time. Multitask learning uses the relationship between these tasks to enhance the clustering performance of a single task [33]. The definition of multitask learning is as follows: Assume learning tasks is **T**={*t*_1_, *t*_2_,…*t*_*T*_,}, all tasks are related but different. Multitask learning is aimed at improving the learning performance of each task by using public knowledge [34]. Multitask learning is applied to natural language processing, disease prediction, computer vision, etc. [35]. The information contained in each task helps other tasks learn better. Because different tasks usually have different noises, learning together will offset some noises to some extent. Multitask learning strategy has better generalization performance than single-task learning. In addition, it has better performance and robustness.

## 3. Brain MRI Images Segmentation Based on Multitask Fuzzy *C*-Means Algorithm

### 3.1. WMT-FCM

FCM is a fuzzy clustering method based on the objective function. Essentially, solving the objective function is an iterative optimization process. Therefore, the algorithm is easily affected by noise and random initialization of cluster centers and falls into a local optimum. In the clustering process, different MRI images have very similar cluster centers. The cluster centroids represent related information of different tasks. This related information helps to converge the objective function and avoids the negative effect of noise in MRI images [18]. It benefits the improvement of cluster analysis. However, the traditional single-task FCM is only suitable for a single-task scenario and exploits limited information. It cannot mine public information between different tasks.

Multitask technology has the advantage of mining public information contained in multiple tasks. To utilize the public information and improve the segmentation performance, we introduce multitask technology into the traditional FCM algorithm. Multitask clustering algorithm enables the collaborative learning of different tasks in the clustering process. It makes maximum use of the data information of each task. Because different segmentation tasks usually have different noises, we cannot directly assign the same weight to each task. The task with a better clustering effect should give a higher contribution to the public information. Therefore, a weighted multitask fuzzy C-means (WMT-FCM) algorithm with adaptive adjustment capability is proposed in this paper.  Figure 1 is the schematic diagram of the WMT-FCM algorithm.

Assuming a dataset contains *T* tasks, and each task has *N*_*t*_ pixels. The objective function is proposed as follows:

(5) $$\begin{array}{c} J_{WMT-FCM}=\overset{T}{\underset{t=1}{\sum }}\overset{N_{t}}{\underset{i=1}{\sum }}\overset{C_{t}}{\underset{j=1}{\sum }}u_{ij,t}^{m}{\left\|x_{i,t}-v_{j,t}\right\|}^{2}+\lambda \overset{T}{\underset{t=1}{\sum }}\overset{D}{\underset{d=1}{\sum }}\overset{C_{t}}{\underset{j=1}{\sum }}w_{d,t}p_{jd,t}^{m}{\left\|v_{j,t}-z_{d}\right\|}^{2}+\gamma \overset{T}{\underset{t=1}{\sum }}\overset{D}{\underset{d=1}{\sum }}w_{d,t}\log\left(w_{d,t}\right)\text{.} \end{array}$$

The objective function constraints are as follows:

(6) $$\begin{array}{c} \left\{\begin{array}{cc} \overset{C_{t}}{\underset{j=1}{\sum }}u_{ij,t}=1\text{,} & 1\leq i\leq N,u_{ij,t}\in \left[0,1\right]\text{,}\\ \overset{D}{\underset{d=1}{\sum }}p_{jd,t}=1\text{,} & 1\leq j\leq C_{t},1\leq t\leq T\text{,}\\ \overset{T}{\underset{t=1}{\sum }}w_{d,t}=1\text{,} & 1\leq d\leq D\text{.} \end{array}\right) \end{array}$$

  Where *x*_*i*,*t*_ is the *i*th data sample of the *t*th task, *v*_*j*,*t*_ is the *j*th private cluster center of the *t*th task, and **Z**={*z*_1_, *z*_2_,…, *z*_*D*_} is the public cluster center vector of all tasks. **U**^(*t*)^=[*u*_*ij*,*t*_]_*C*_*t*_×*N*_*t*__ is the private membership matrix of the *t*th task. *p*_*jd*,*t*_ represents the membership value of private cluster center *v*_*j*,*t*_ to the *d*th public cluster center *z*_*d*_. *D* is the number of public cluster centers. *λ* is a balance parameter to control the influence of the public clustering term. *γ* is used to adjust the penalty corresponding to the weights of each task. **W**^(*t*)^={*w*_1,*t*_, *w*_2,*t*_,…, *w*_*D*,*t*_} is the weight vector of the *t*th task. *w*_*d*,*t*_ represents the importance of the *t*th task to the *d*th public cluster.

The first part of the objective function contains *T*-independent FCM clustering tasks. The first part aims to learn the within-task partition matrix and cluster centers. The second part aims to learn public information about all tasks. It uses the FCM objective function to learn the public partition matrix and public cluster centers. The third part is the regularization term. We introduce the Shannon entropy as the regularizer. The third part aims to identify the optimal weights of each task.

Although there is public information about different tasks, the difference also exists between all tasks. For example, each task is affected by varying levels of noise and has different clustering effectiveness. Therefore, the influence of different tasks should be adjusted according to the actual situation instead of keeping it consistent. Considering the difference between separate tasks, we introduce the adaptive weight *w*_*d*,*t*_. *w*_*d*,*t*_ controls the impact of the *t*th task on the *d*th public cluster centers. If the relationship is clearer between the private cluster centers and the public clustering centers, a higher weight value is given. That means the task has a greater contribution to the public cluster centers. Conversely, if the relationship is fuzzier with public cluster centers, a lower weight parameter is given. The algorithm can utilize the effective public information of different tasks to the greatest extent and improve the clustering performance through adaptive weight adjustment.

### 3.2. Optimization

The Lagrange multiplier method is used to obtain the minimization of equation (5). According to the corresponding constraints, the objective Lagrangian function is defined as follows:

(7) $$\begin{array}{c} J_{WMT-FCM}=\overset{T}{\underset{t=1}{\sum }}\overset{N_{t}}{\underset{i=1}{\sum }}\overset{C_{t}}{\underset{j=1}{\sum }}u_{ij,t}^{m}{\left\|x_{i,t}-v_{j,t}\right\|}^{2}+\lambda \overset{T}{\underset{t=1}{\sum }}\overset{D}{\underset{d=1}{\sum }}\overset{C_{t}}{\underset{j=1}{\sum }}w_{d,t}p_{jd,t}^{m}{\left\|v_{j,t}-z_{d}\right\|}^{2}+\gamma \overset{T}{\underset{t=1}{\sum }}\overset{D}{\underset{d=1}{\sum }}w_{d,t}\log\left(w_{d,t}\right)+\overset{T}{\underset{t=1}{\sum }}\overset{N_{t}}{\underset{i=1}{\sum }}a_{i,t}\left(1-\overset{C_{t}}{\underset{j=1}{\sum }}u_{ij,t}\right)+\overset{T}{\underset{t=1}{\sum }}\overset{C_{t}}{\underset{j=1}{\sum }}b_{j,t}\left(1-\overset{D}{\underset{d=1}{\sum }}p_{jd,t}\right)+\overset{D}{\underset{d=1}{\sum }}c_{d}\left(1-\overset{T}{\underset{t=1}{\sum }}w_{d,t}\right)\text{,} \end{array}$$

where *a*_*i*,*t*_, *b*_*j*,*t*_, and *c*_*d*_ are the Lagrange multipliers corresponding to the constraints (∀i ∈ {1,2,…, *N*_*t*_}, ∀j ∈ {1,2,…, *C*_*t*_}, ∀*d* ∈ {1,2,…, *D*}, ∀*t* ∈ {1,2,…, *T*}).

#### 3.2.1. Optimizing Membership Matrix

Taking the derivative of *J*_WMT−FCM_ with respect to *u*_*ij*,*t*_ and setting it to zero, we obtain

(8) $$\begin{array}{c} \frac{\partial J_{WMT-FCM}}{\partial u_{ij,t}}=u_{ij,t}^{m-1}{\left\|x_{i,t}-v_{j,t}\right\|}^{2}-a_{i,t}.\\ =0\text{.} \end{array}$$

From equation (8), *u*_*ij*,*t*_ is calculated as follows:

(9) $$\begin{array}{c} u_{ij,t}=\frac{{a_{i,t}}^{1/m-1}}{{\left({\left\|x_{i,t}-v_{j,t}\right\|}^{2}\right)}^{1/m-1}}\text{.} \end{array}$$

According to ∑_*l*=1_^*C*_*t*_^*u*_*il*,*t*_=1 and equation (9), *a*_*i*,*t*_ can be obtained as follows after the necessary calculations:

(10) $$\begin{array}{c} a_{i,t}=\frac{1}{{\left[\overset{C_{t}}{\underset{l=1}{\sum }}{\left({\left\|x_{i,t}-v_{l,t}\right\|}^{2}\right)}^{-1/m-1}\right]}^{1/m-1}}\text{.} \end{array}$$

By substituting equation (10) into equation (9), the iterative formulate of private membership value *u*_*ij*,*t*_ for *t*th task is as follows:

(11) $$\begin{array}{c} u_{ij,t}=\frac{{\left({\left\|x_{i,t}-v_{j,t}\right\|}^{2}\right)}^{-\left(1/m-1\right)}}{\sum_{l=1}^{C_{t}}{\left({\left\|x_{i,t}-v_{j,t}\right\|}^{2}\right)}^{-\left(1/m-1\right)}}\text{.} \end{array}$$

Similarly, the updating equation of the membership value *p*_*jd*,*t*_ is as follows:

(12) $$\begin{array}{c} p_{jd,t}=\frac{{\left({w_{d,t}\left\|v_{j,t}-z_{d}\right\|}^{2}\right)}^{-\left(1/m-1\right)}}{\sum_{l=1}^{D}{\left({w_{l,t}\left\|v_{j,t}-z_{l}\right\|}^{2}\right)}^{-\left(1/m-1\right)}}\text{.} \end{array}$$

#### 3.2.2. Optimizing Cluster Centroid

Taking the derivative of *J*_WMT−FCM_ with respect to *v*_*j*,*t*_ and setting it to zero, we obtain

(13) $$\begin{array}{c} \frac{\partial J_{WMT-FCM}}{\partial v_{j,t}}=-\overset{N_{t}}{\underset{i=1}{\sum }}u_{ij,t}^{m}\left(x_{i,t}-v_{j,t}\right)+\lambda \overset{D}{\underset{d=1}{\sum }}w_{d,t}p_{jd,t}^{m}\left(v_{j,t}-z_{d}\right)\\ =0\text{.} \end{array}$$

According to equation (13), private clustering centroid *v*_*j*,*t*_ is obtained as following after necessary calculations:

(14) $$\begin{array}{c} v_{j,t}=\frac{\sum_{i=1}^{N_{t}}u_{ij,t}^{m}x_{i,t}+\lambda \sum_{d=1}^{D}w_{d,t}p_{jd,t}^{m}z_{d}}{\sum_{i=1}^{N_{t}}u_{ij,t}^{m}+\lambda \sum_{d=1}^{D}w_{d,t}p_{jd,t}^{m}}\text{.} \end{array}$$

Similarly, the updating equation of the public clustering centroid *z*_*d*_ is as follows:

(15) $$\begin{array}{c} z_{d}=\frac{\sum_{t=1}^{T}\overset{C_{t}}{\underset{j=1}{\sum }}w_{d,t}p_{jd,t}^{m}v_{j,t}}{\sum_{t=1}^{T}\overset{C_{t}}{\underset{j=1}{\sum }}w_{d,t}p_{jd,t}^{m}}\text{.} \end{array}$$

#### 3.2.3. Optimizing Weight

To derive the optimal weights, taking the derivative of the Lagrangian function with respect to *w*_*d*,*t*_ and setting it to zero as follows:

(16) $$\begin{array}{c} \frac{\partial J_{WMT-FCM}}{\partial w_{d,t}}=\lambda \sum_{j=1}^{C_{t}}p_{jd,t}^{m}{\left\|v_{j,t}-z_{d}\right\|}^{2}+\gamma \left(1+\ln w_{d,t}\right)-c_{d}\\ =0\text{.} \end{array}$$

According to ∑_*t*=1_^*T*^*w*_*d*,*t*_=1 and equation (16), we can obtain the optimal weight *w*_*d*,*t*_ using steps similar to optimize the membership matrix as follows:

(17) $$\begin{array}{c} w_{d,t}=\frac{\exp\;\left(-\lambda \overset{C_{t}}{\underset{j=1}{\sum }}p_{jd,t}^{m}{\left\|v_{j,t}-z_{d}\right\|}^{2}/\gamma \right)}{\overset{T}{\underset{h=1}{\sum }}\exp\;\left(-\lambda \overset{C_{t}}{\underset{j=1}{\sum }}p_{jd,t}^{m}{\left\|v_{j,t}-z_{d}\right\|}^{2}/\gamma \right)}\text{.} \end{array}$$

The specific steps of WMT-FCM are summarized in Algorithm 1.

## 4. Experimental Results

### 4.1. The Experimental Dataset

To demonstrate the improvement of the proposed algorithm, the traditional FCM and DMFCM [18] are selected as comparison algorithms. The dataset of this study is downloaded from BrainWeb. The BrainWeb is acquired from the McConnell Brain Imaging Center of the Montreal Neurological Institute, McGill University [36]. This database contains a set of realistic MRI data produced by an MRI simulator. The BrainWeb simulates 3-dimensional data volumes using three sequences (*T*1, *T*2, and PD weighted). The simulated volumes contain a variety of slice thicknesses, noise levels, and intensity nonuniformity (INU) levels. The ground truth of the cerebral spinal fluid (CSF), the gray matter (GM), the white matter (WM), and the background are available.

The BrainWeb dataset in our work consists of 9 *T*1-weighted MRI images (slice 90) with 181217 pixels. The MRI images are corrupted with different levels of noise and INU. Details are shown in Table 2. These images are randomly combined as task groups. The ground truth images of the brain MRI images are shown in Figure 2.

### 4.2. Parameters Setting

*λ* and *γ* of the objective function influence the cluster centers and weight vectors according to equations (8) and (11). In this study, the optimal parameters of the proposed algorithm are obtained by the grid search strategy. *λ* and *γ* are set from two grids {20, 40, 60, 80,100, 120} and {0.2, 0.4, 0.6, 0.8, 1, 1.2}, respectively. In addition, all experiments are conducted with the maximum number of iterations *K* = 100, termination parameter *ε*=0.0001, cluster index *m* = 2.

### 4.3. Evaluation Index

The quantitative performance comparison is performed using the Dice similarity coefficient (DSC) [37] and segmentation accuracy (SA) [38].

*(1) Dice Similarity Coefficient*. DSC measures the similarity between the ground truth and segmentation results. According to equation (12), *S*_1_ represents the segmentation results. *S*_2_ represents the ground truth for a single class. Here the DSC measures the similarity of CSF, GM, WM, and background. The larger value of DSC indicates the better performance of the algorithm.

(18) $$\begin{array}{c} DSC=\frac{2\left|S_{1}\cap S_{2}\right|}{\left|S_{1}\right|+\left|S_{2}\right|}\text{.} \end{array}$$

*(2) Average Dice Similarity Coefficient*. The average Dice similarity coefficient [39] of WM, GM, and CSF is described as equation (13). Considering the nonbrain tissue background, we exclude it during the average DSC (DSC_av_) calculating.

(19) $$\begin{array}{c} {DSC}_{av}=\frac{2\left(\left|S_{1}^{CSF}\cap S_{2}^{CSF}\right|+\left|S_{1}^{GM}\cap S_{2}^{GM}\right|+\left|S_{1}^{WM}\cap S_{2}^{WM}\right|\right)}{\left|S_{1}^{CSF}\right|+\left|S_{2}^{CSF}\right|+\left|S_{1}^{GM}\right|+\left|S_{2}^{GM}\right|+\left|S_{1}^{WM}\right|+\left|S_{2}^{WM}\right|}\text{.} \end{array}$$

*(3) Segmentation Accuracy*. SA index measures the accuracy of the algorithm. Given in equation (14), where *A*_*i*_ is the pixel set of the *i*th cluster belonging to segmented results, *B*_*i*_ is the pixel set belongs to ground truth, and *K* is the number of clusters. The closer SA to 1 indicates better segmentation performance. The evaluation metric is defined as follows:

(20) $$\begin{array}{c} SA=\frac{\overset{C}{\underset{i=1}{\sum }}A_{i}\cap B_{i}}{\overset{C}{\underset{l=1}{\sum }}B_{l}}\text{.} \end{array}$$

The metrics are an average of ten repeated experiments since the performance of FCM depends on the random initialization of the cluster centroids. Select 3 images with different levels of noise and intensity nonuniformity as a task group randomly. The inputs are segmented into the following four clusters: background, CSF, GM, and WM. All experiments are conducted on MATLAB 2019a and executed with a PC configured with a 1.50 GHz CPU and 16G memory Intel Core i7 processor, Windows 10.

## 5. Results and Discussion

To verify the stability and the antinoise ability improvement of the WMT-FCM algorithm, this section gives a comparison with classical FCM and DMFCM. There are nine MRI images from BrainWeb, as shown in Table 2.

Figure 3 shows the original images of 9 simulated MRI brain images (slice 90) as well as the corresponding segmentation results of the WMT-FCM algorithm. Segmented images include the entire image and individual tissues. Figure 2 displays the ground truth images of simulated MRI images (slice 90). Figure 3 qualitatively reveals that the WMT-FCM algorithm could partition different tissues. The segmented images overlap well with the ground truth on all tested images.

Table 3 shows the experimental results of the following three different algorithms: FCM, DMFCM, and the proposed WMT-FCM. The results include the mean values of the SA, DSC_av_ of all tissues. The WMT-FCM segmentation performance is significantly better than FCM. This shows It confirms that the introduction of multitask learning mechanism mines public information from multiple tasks. Compared with DMFCM, the segmentation effect of the WMT-FCM algorithm in this study is better. This demonstrates the effectiveness of the task weight learning mechanism. To archive the results, the single task execution time of FCM, WMT-FCM, and DMFCM is about 1 second, 6 seconds, and 600 seconds. The execution time of multitask algorithms is higher than classical FCM since the public partition matrix and the public cluster center learning require more time. However, even if the execution time is increased, the execution time of the WMT-FCM algorithm is still much shorter than DMFCM.

To further compare segmentation performance, the Dice similarity coefficient of each tissue is calculated. The result is presented in Table 4. WMT-FCM provides better results than FCM and DMFCM in WM, GM, and CSF generally. Among the three tissues, the performance of WMT-FCM is the best in WM and relatively poor in GM. However, even though the WMT-FCM segmentation performance is slightly inferior in GM. It is still significantly superior to FCM and DMFCM. FCM and DMFCM always fail to distinguish CSF accurately.

### 5.1. Robustness to Noise

Figure 4 shows SA and DSC_av_ of the algorithms on the images with 20% INU and different noise levels. As the images with a higher noise level, the clustering performance of both clustering algorithms is lower. The WMT-FCM clustering performance is better than the comparison algorithms, even if each algorithm's performance is declining with the noise level increasing. In addition, with the noise increasing, the WMT-FCM clustering performance decreases less than FCM and DMFCM, which indicates that WMT-FCM is more robust to noise.

### 5.2. Sensitivity to Initialization

Figure 5 displays the SA variations in repeated trials on image 3. The SA of FCM changed dramatically in different trials. Since the initialization of the clustering centroids is random, the FCM clustering performance depends on the initial values of cluster centers. Therefore, the results of the fuzzy clustering-based algorithm are usually inconsistent in repeated trials. However, the segmentation results of WMT-FCM are almost unchanged. In addition, SA values of WMT-FCM are higher than FCM and DMFCM in almost all trials. Repeated trials indicate that WMT-FCM is more robust to the initialization compared with FCM and DMFCM and generates consistent excellent segmentation performance.

To compare the algorithms' performance more visually, the visual results are shown in Figures 6 and 7.  Figure 6 displays the segmented images of the first to fourth trials on image 3 by FCM, DMFCM, and WMT-FCM. FCM fails to partition the brain tissues in almost all trials, especially CSF, except the third trial. In the first trial, all tissues are segmented as an individual cluster, background. In the second trial, FCM drops the CSF region and oversegmented GM. FCM shows a relatively good result in the third trial. In the fourth trial, FCM fails to detect CSF as well as GM and oversegmented the WM. DMFCM always tends to lose CSF. However, in the four trials, WMT-FCM offers an excellent overlap with ground truth consistently. A detailed comparison is shown in Figure 7, which indicates the proposed algorithm has superior segmentation performance than FCM, especially on GM and CSF. It can be concluded that the WMT-FCM algorithm provides better performance consistently and is less sensitive to the random initialization.

### 5.3. Sensitivity to Parameters

The experiments explore the sensitivity of the WMT-FCM parameters are conducted. The crucial parameters, i.e., the balance parameter *λ* and regularization coefficients *γ* are involved.  Figure 8 shows the sensitivity of parameters with respect to the two different MRI images (image 4 and image 6). WMT-FCM provides relatively excellent segmentation results when the core parameters are located within the proper interval. Overall, the algorithm performance is slightly sensitive to the parameters, especially on DSC_av_. The algorithm is more sensitive to trade-off parameter *λ* than the corresponding regularization parameter *γ*. Therefore, *λ* plays a major role in obtaining optimal clustering results. With the *λ* increasing, the segmentation performance of image 4 (with 1% noise and no INU) shows a decreasing trend. Image 6 (with 9% noise and 20% INU) shows a tendency to rise first and fall after. Excessive trade-off parameter enhances the influence of public information on clustering results and leads to undesirable effects. The performance may decrease, especially on images with a low level of noise and INU. In summary, although the proposed algorithm is slightly sensitive to trade-off parameter *λ*, it obtains relatively good performance within an appropriate range.

## 6. Conclusions

In this paper, we propose a new fuzzy clustering algorithm called WMT-FCM. Multitask learning mechanism is introduced into the FCM algorithm for brain MRI image segmentation. WMT-FCM makes use of both private information in a single task and public information among related tasks. To draw more effective public information from different tasks, we design an adaptive task weighting mechanism. We take experiments to validate the proposed algorithm on synthetic MRI images. The results demonstrate that the proposed algorithm provides more accurate segmentation results than the FCM and DMFCM algorithms. WMT-FCM has the following advantages: (1) WMT-FCM is less sensitive to the initialization of cluster centers; (2) the robustness to noise is improved; (3) WMT-FCM is adaptive to the private clustering effect. There are two main limitations in the WMT-FCM. The algorithm requires more computational time for public information learning and adaptive weights updating. Although the proposed algorithm obtains a relatively good effect when the trade-off parameter *λ* is in the appropriate range, the performance is slightly sensitive to *λ*. In later research, we will focus on how to tackle these problems. In conclusion, the algorithm based on FCM and multitask learning significantly improves the segmentation performance of brain MRI images. The main limitations of the FCM algorithm, that is, the sensitivity to initialization and noise have been partially improved.

## Figures and Tables

**Figure 1:** The schematic diagram of the WMT-FCM algorithm.

**Figure 2:** Ground truth images of the simulated brain MRI images: (a) total; (b) WM; (c) GM; (d) CSF.

**Figure 3:** Segmentation results of simulated MRI brain images (slice 90) with different noises and INU in the WMT-FCM algorithm.

**Figure 4:** The variations of SA and average DSC on images with 20% INU and increasing noise level by FCM, DMFCM, and WMT-FCM: (a) SA and (b) DSC_av_.

**Figure 5:** SAvariations of FCM, DMFCM, and WMT-FCM on image 3 in repeated trials.

**Figure 6:** Segmentation results on image 3 in repeated trials (trials 1, 2, 3, and 4). The black image indicates all tissues are segmented as one cluster (background).

**Figure 7:** Comparison of segmentation results on image 3 in trial 2 between FCM, DMFCM, and WMT-FCM. The black image indicates FCM fails to detect the CSF.

**Figure 8:** Average SA and DSC_av_ of WMT-FCM on image 4 and image 6 with trade-off parameter *λ* and corresponding regularization parameter *γ*: (a) SA vs. *λ*; (b) SA vs. *γ*; (c) DSC_av_ vs. *λ*; (d) DSC_av_ vs. *γ*.

**Algorithm 1:** WMT-FCM.

**Table 1:** Description of symbols in FCM.

Symbol	Description
**X**	Input dataset
**V**	Cluster centers vector
**U**	Membership matrix
*C*	Number of the clusters
*N*	Total number of samples
*x*_*i*_	The *i*th sample
*v*_*j*_	The *j*th cluster center
*u*_*ij*_	The membership degree of *x*_*i*_ to *v*_*j*_
*M*	Fuzzy factor

**Table 2:** Information about the simulated MRI images.

	Image 1 (%)	Image 2 (%)	Image 3 (%)	Image 4 (%)	Image 5 (%)	Image 6 (%)	Image 7 (%)	Image 8 (%)	Image 9 (%)
Noise	1	5	7	1	7	9	3	3	5
INU	20	20	0	0	20	20	20	0	0

**Table 3:** The average values in terms of segmentation accuracy and average Dice similarity coefficient on simulated MRI brain images.

Image	SA			DSC_av_		
	FCM	DMFCM	WMT-FCM	FCM	DMFCM	WMT-FCM
Image 1	0.8943	0.9531	0.9870	0.8059	0.9230	0.9737
Image 2	0.8668	0.9131	0.9705	0.7425	0.8366	0.9408
Image 3	0.8289	0.8765	0.9537	0.6705	0.7716	0.9081
Image 4	0.9142	0.9630	0.9914	0.8469	0.9390	0.9826
Image 5	0.8268	0.8686	0.9543	0.6752	0.7541	0.9090
Image 6	0.7979	0.8618	0.9237	0.6107	0.7415	0.8495
Image 7	0.8781	0.9164	0.9818	0.7789	0.8521	0.9632
Image 8	0.8905	0.8865	0.9845	0.8089	0.7932	0.9688
Image 9	0.8712	0.8778	0.9737	0.7572	0.7677	0.9472

**Table 4:** The average values in terms of the Dice similarity coefficient for a single tissue, including WM, GM, and CSF.

Image	WM			GM			CSF		
	FCM	DMFCM	WMT-FCM	FCM	DMFCM	WMT-FCM	FCM	DMFCM	WMT-FCM
Image 1	0.8989	0.9791	0.9801	0.6555	0.9317	0.9649	0.3901	0.4876	0.9750
Image 2	0.7425	0.9064	0.9550	0.6327	0.7248	0.9219	0.4716	0.5657	0.9424
Image 3	0.7708	0.8851	0.9309	0.5067	0.6615	0.8793	0.2717	0.1815	0.9060
Image 4	0.9303	0.9852	0.9887	0.7525	0.9454	0.9769	0.3915	0.5872	0.9772
Image 5	0.8207	0.8649	0.9306	0.4161	0.5926	0.8818	0.0910	0.2729	0.9090
Image 6	0.7317	0.8583	0.8885	0.3946	0.6271	0.8089	0.1662	0.1662	0.8316
Image 7	0.8933	0.9414	0.9729	0.6328	0.8051	0.9508	0.1927	0.2891	0.9628
Image 8	0.9232	0.8967	0.9773	0.7225	0.6457	0.9583	0.0968	0.2903	0.9672
Image 9	0.8367	0.8375	0.9616	0.7061	0.7137	0.9297	0.2838	0.3784	0.9440

## Data Availability

The public datasets used to validate the study can be obtained from BrainWeb (https://brainweb.bic.mni.mcgill.ca/brainweb/).
